# A Systematic Review on the Management of Transfusion-Related Acute Lung Injury in Transfusion-Dependent Sickle Cell Disease

**DOI:** 10.7759/cureus.22101

**Published:** 2022-02-10

**Authors:** Hadia Arzoun, Mirra Srinivasan, Mona Adam, Siji S Thomas, Bridget Lee, Alena Yarema

**Affiliations:** 1 Internal Medicine, California Institute of Behavioral Neurosciences & Psychology, Fairfield, USA; 2 Internal Medicine, St. Bernards Medical Center, Jonesboro, USA

**Keywords:** current guidelines, complications, management, sickle cell disease, transfusion-related acute lung injury

## Abstract

The onset of respiratory distress and acute lung injury (ALI) following a blood transfusion is known as transfusion-related acute lung injury (TRALI), although its pathophysiology remains unknown. Even though sickle cell disease (SCD) has been studied for more than a century, few therapeutic and management strategies adequately address the emergence of TRALI. TRALI, an immune-mediated transfusion response that can result in life-threatening consequences, is diagnosed based on clinical signs and symptoms. Early detection and treatment increase the chances of survival and, in most cases, result in a complete recovery. Our objective is to provide a firm grasp of the present status of SCD-related TRALI care and therapy.

After exploring multiple databases, this study offers evidence-based guidelines to aid clinicians and other healthcare professionals make decisions concerning transfusion assistance for SCD and the management of transfusion-related complications. Other risk factors for acute lung injury including sepsis aspiration should be ruled out throughout the diagnostic process. Several recent studies have shown that immunotherapy or immunological targets can effectively prevent these complications. Red cell transfusions, red cell antigen matching optimization, and iron chelation can also help reduce negative consequences. It is to be noted that poor clinical outcomes can be avoided by early detection and treatment of hemolytic transfusion reactions. Finally, preventing the onset of TRALI may be the most effective therapeutic strategy for SCD patients who rely on blood transfusions for survival.

## Introduction and background

Sickle cell disease (SCD) is a disease in which the appearance of red blood cells takes on the shape of a sickle [1]. The condition causes the breakdown of red blood cells prematurely, resulting in anemia. Due to their deformed shape, sickle cells tend to become trapped within small vessels and deprive the tissues of blood that is rich in oxygen [2]. The onset of SCD is often accompanied by various complications, including hemolytic anemia, reduced immunity, inflammation, acute/chronic organ damage, and stroke, among others [3]. Therefore, providing effective treatment to patients impacted by SCD is critical. However, common treatment protocols, such as blood transfusions, can result in complications and adverse effects, particularly among those dependent on transfusions [4]. The emergence of transfusion-related acute lung injury (TRALI) [5], which is defined as acute pulmonary edema following transfusion in the absence of circulatory overload or other acute respiratory distress syndrome (ARDS) risk factors [6], is a major complication associated with blood transfusion in SCD patients. The total number of blood products administered, independent of component type, and cardiac dysfunction with signs of elevated filling pressures, leading to pulmonary edema, are other transfusion-specific risk factors for TRALI [6]. Therefore, transfusion-dependent patients are at an increased risk for TRALI. Due to the serious nature of TRALI related to SCD, management and treatment options have been sought. However, treatment and management options primarily revolve around supportive care modalities and preventative measures. Supportive care often includes oxygen supplementation, mechanical ventilation, albumin treatment, and the provision of erythropoietin and iron supplementation [5,7-9]. Preventative measures that are being employed and explored include blood antibody testing of donors, enhanced and standardized blood and plasma selection protocols, rapid reporting to blood banks, and rituximab prophylaxis [5,8-10]. Finally, due to limited effective treatment modalities, the use of the anti-CD40L monoclonal antibody, as well as immunotherapy, is being studied as a potential option in the future [11,12]. The purpose of this review article is to explore each of these aspects and summarize the current state of SCD-related TRALI management and treatment.

Methodology

This systematic review follows the Preferred Reporting Items for Systematic Reviews and Meta-Analysis (PRISMA) 2020 guidelines and principles [13]. The Boolean technique with medical subject headings (MeSH) was employed in PubMed, and regular keywords were employed in other databases, namely, Google Scholar and Science Direct. This search yielded a total of 488 articles, of which 36 were duplicates, 452 were retrieved for screening, 358 were excluded based on the titles and abstracts, and 48 were excluded based on the exclusion criteria. Nine reports were selected as the final studies after undergoing quality assessments which were done separately by two authors. In cases of discrepancies among the authors, a third author was approached to find common ground. The search strategy and the process of selecting the final studies are depicted in Figure 1 below in the form of a PRISMA flowchart [13].

**Figure 1:** PRISMA flowchart 2020. PRISMA: Preferred Reporting Items for Systematic Reviews and Meta-Analysis

The inclusion and exclusion criteria set for this study are depicted in Table 1 below.

**Table 1:** Inclusion and exclusion criteria.

Inclusion	Exclusion
Studies from the past six years	Studies prior to 2015
Full-text studies	Non-Full text, only abstract studies
English-language studies	Studies in languages other than English
Worldwide studies	Specific geographical location
Study designs such as review articles, and animal studies	Other study designs

The regular and MeSH keywords used for this study are depicted in Table 2 below.

**Table 2:** Keywords employed in this study. MeSH: medical subject headings

	Keywords used
Regular keywords	Transfusion-related acute lung injury; sickle cell disease; management; complications; current guidelines
MeSH keywords	Transfusion-related acute lung injury OR ((“Transfusion-Related Acute Lung Injury/blood”[Mesh] OR “Transfusion-Related Acute Lung Injury/classification”[Mesh] OR “Transfusion-Related Acute Lung Injury/complications”[Mesh] OR “Transfusion-Related Acute Lung Injury/diagnosis”[Mesh] OR “Transfusion-Related Acute Lung Injury/etiology”[Mesh] OR “Transfusion-Related Acute Lung Injury/immunology”[Mesh] OR “Transfusion-Related Acute Lung Injury/mortality”[Mesh] OR “Transfusion-Related Acute Lung Injury/physiopathology”[Mesh] OR “Transfusion-Related Acute Lung Injury/prevention and control”[Mesh] OR “Transfusion-Related Acute Lung Injury/therapy”[Mesh])) AND Sickle cell disease OR (“Anemia, Sickle Cell/complications”[Mesh] OR “Anemia, Sickle Cell/diagnosis”[Mesh] OR “Anemia, Sickle Cell/drug therapy”[Mesh] OR “Anemia, Sickle Cell/immunology”[Mesh] OR “Anemia, Sickle Cell/metabolism”[Mesh] OR “Anemia, Sickle Cell/physiopathology”[Mesh] OR “Anemia, Sickle Cell/prevention and control”[Mesh] OR “Anemia, Sickle Cell/therapy”[Mesh])

Results

Table 3 provides a summary of the characteristics of the final included studies for this review article [4,8-12,14-16].

**Table 3:** Summary of characteristics of the final included studies. SANRA: A Scale for the Quality Assessment of Narrative Review Articles; HLA: human leukocyte antigens; FFP: fresh frozen plasma; PAS: platelet additive solutions; TRALI: transfusion-related acute lung injury; ALI: acute lung injury; IL: interleukin; SYCRLE: Systematic Review Center for Laboratory Animal Experimentation; DHTR: delayed hemolytic transfusion reactions; SCD: sickle cell disease; Rh: Rhesus; PRISMA: Preferred Reporting Items for Systematic Reviews and Meta-Analysis; TACO: transfusion-associated circulatory overload

Author	Year	Type of study	Quality appraisal tool	Conclusions
Kim and Na [8]	2015	Review article	SANRA Checklist	Four takeaways: (1) The decision to transfuse should take into account the patient’s clinical condition, co-morbidities, and individual wishes; (2) donors with a low chance of alloimmunization to leukocytes should receive high plasma volume components; (3) Use pooled solvent detergent-treated plasma as an alternative to FFP; and (4) before apheresis of platelets or plasma, test for anti-HLA antibodies in pregnant donors
Otrock et al. [10]	2017	Review article	SANRA Checklist	When used in conjunction with existing mitigation methods, new procedures such as HLA antibody screening, PAS, and washing can significantly lower TRALI risk. To avoid transfusions when not needed, physicians should pay close attention to the patient’s risk factors for ALI and use evidence-based transfusion protocols
Semple et al. [4]	2018	Review article	SANRA Checklist	IL-10 therapies, lowering C-reactive protein levels, targeting reactive oxygen species, and inhibiting IL-8 receptors are all viable therapeutic methods for the transfused recipient
Raja et al. [9]	2019	Review article	SANRA Checklist	TRALI can be diagnosed earlier if clinicians are aware of the disorder and have a high index of suspicion. Other risk factors for ALI, such as sepsis and aspiration, should be ruled out during the diagnostic process. TRALI is treated the same way as ALI, with symptomatic and supportive care
Tariket et al. [12]	2019	Animal atudy	SYRCLE’s Assessment Tool	To reduce the risk of TRALI, data show that improving the conditions in which platelet concentrates are manufactured and kept at lower sCD40L levels is critical. Preventative and curative therapies can be proposed with a better understanding of the first TRALI hit along with patient’s risk factors. Identification of patients at risk for TRALI will allow for proactive, customized therapy, resulting in better patient care
Guo and Ma [11]	2021	Review article	SANRA Checklist	Innate immune molecules, such as complement, are also significant, while IL-10 treatment is a viable therapeutic method to investigate further
Linder and Chou [14]	2021	Review article	SANRA Checklist	Because of the complications of iron overload, alloimmunization, and DHTR, transfusion should only be done for evidence-based or expert-defined purposes. High rates of alloimmunization continue despite a greater understanding of the pathophysiology of alloimmunization in SCD and improved Rh and K antigen matching. Future research is needed to see if preventive Rh genotype matching or extended antigen matching can cost-effectively minimize alloimmunization
Van den Akker et al. [15]	2021	Review article	SANRA Checklist	The understanding and awareness of TACO risk factors, possible TRALI primed situations, and ARDS risk factors are critical for clinicians and treating medical professionals. With a greater understanding that TACO or TRALI is more likely to occur in specific situations, early recognition and reporting can occur if it happens
Hu et al. [16]	2021	Review (systematic) article	PRISMA Checklist	The findings imply that host-related risk factors are more relevant than blood transfusion-related risk factors in the onset and progression of TRALI

## Review

This section provides a comprehensive understanding of SCD along with its complications, the treatment protocols, risk factors, and TRALI-related complications, as well as the management of these complications, ending with a note on potential future treatments.

Background and significance

First identified in 1910, SCD presented as a mysterious condition that disproportionately affected people of color and was considered as one of the most common hereditary diseases globally. In the United States, SCD affects approximately 80,000-100,000 individuals [1]. Globally, an estimated 300,000 children are affected. Researchers and hematologists continue to express their concerns regarding the lack of effective treatment options available for SCD and the need to advance treatment modalities in addition to supportive care practices [1].

There are several complications associated with SCD. Serious complications include the onset of acute chest syndrome (ACS), avascular necrosis, hemolytic anemia, silent cerebral infarction, inflammation, priapism, and stroke. Moreover, serious complications often revolve around organ damage, eventually resulting in organ failure, including renal failure [2,3]. Apart from the disease complications, treatment-related adverse effects also occur, especially in those who require frequent blood transfusions, most commonly presenting as TRALI [5]. To enhance the health and life span of these individuals, complications associated with the disease and treatment require effective management strategies.

A note on transfusion-dependent acute lung injury

TRALI refers to the onset of acute lung injury caused by blood transfusions that result in respiratory distress [11]. The onset of TRALI often causes hemodynamic instability and presents with symptoms, such as tachycardia, hypotension, and fever. In some cases, the peripheral neutrophil count may also be decreased [17]. Other common symptoms include nausea, vomiting, and anaphylaxis [15]. TRALI often presents with pulmonary lesions and immune cell infiltration in the alveolar space [12]. Though similar to transfusion-associated circulatory overload (TACO), TRALI has a few distinguishing characteristics, such as hypotension versus hypertension, lack of widened pulse pressure, exudate pulmonary edema fluid, balanced fluids, and minimal response to diuretics [15]. In the past, TRALI was misdiagnosed or underdiagnosed as a complication related to blood transfusion [6,11,15]. Identifying its presence and distinguishing it from TACO is key to selecting appropriate management and treatment options. Figure 2 depicts the differentiating characteristics of TRALI and TACO [6].

**Figure 2:** TRALI versus TACO. Figure created by the authors on Microsoft PowerPoint. TRALI: transfusion-related acute lung injury; TACO: transfusion-associated circulatory overload; EF: ejection fraction; BNP: brain natriuretic peptide; JVP: jugular venous pressure; B/L: bilateral

Risk factors associated with TRALI are important to consider for treatment, management, and prevention. One major risk factor includes the number of transfusions an individual receives. Moreover, the number of units of fresh frozen plasma for transfusion also increases the risk of TRALI [16]. Other potential risk factors may include female sex, age, chronic alcohol abuse, and tobacco use, among others. Host-related risk factors are believed to play a large role as opposed to blood transfusion factors [16]. Importantly, patients with SCD are at an increased risk of red blood cell alloimmunization, which significantly contributes to the onset of TRALI [5].

Current treatment protocols

Treatment protocols for SCD vary and are undergoing advancements. One treatment that is often provided includes hydroxyurea to address hemoglobin S polymerization. Vaso-occlusion is often addressed using L-glutamine, crizanlizumab, heparinoids, poloxamer, and vepoloxamer. Inflammation has been addressed using prasugrel, intravenous immunoglobulin, simvastatin, rivaroxaban, and N-acetylcysteine. Moreover, the use of allogenic bone marrow transplants has also increased in therapeutic utilization [18]. In more recent treatment attempts, stem cell transplants have been in clinical trials to change the genotype of SCD. This includes gene therapy and gene editing strategies as well [18]. Finally, in cases where signs of circulatory failure are present, red cell transfusions are employed [3]. Traditionally, red cell transfusions have been a common treatment for those with SCD, despite the side effects involved [14,18]. This is due to the ability of blood transfusions to enhance the oxygen-carrying capacity of red blood cells [14]. In many cases, transfusion dependency can occur which increases the number of transfusions SCD patients receive in their lifetime [1,3]. However, transfusion dependency is not ideal as a primary treatment and management modality.

TRALI management options

Management and treatment options for TRALI are relatively limited. This is particularly true for SCD patients who are transfusion-dependent because their underlying condition requires continued transfusion treatments [19]. Currently, all treatment and management protocols are supportive in nature. Moreover, much of the management options focus on preventative measures due to a lack of effective treatment options. However, there are treatments currently in research and clinical trials which attempt to fill the present gap in treatment and management options. Each of these is discussed in the following sections.

Supportive care modalities

As previously mentioned, supportive care therapies are the main form of treatment and management for TRALI. These include oxygen supplementation, mechanical ventilation, albumin treatment, and erythropoietin and iron supplementation.

Oxygen Supplementation

Oxygen supplementation is a primary treatment option to manage the primary result of TRALI, which includes respiratory distress [7-9]. Oxygen is often administered when the breathing becomes labored and the oxygen saturation on room air begins to decrease [7,9]. Acute respiratory failure is often noted when the partial pressure of arterial oxygen (PaO_2_) becomes less than or equal to 8 kPA on room air [7]. This often indicates oxygen is required as supportive care.

Mechanical Ventilation

In approximately 79-90% of cases requiring oxygen, mechanical ventilation is required [9]. This often involves the use of restrictive tidal volume ventilation [8,9]. Signs of hypoxia are identified when the patient’s oxygen saturation decreases to or drops below 94% with oxygen [7]. This process can assist the patient with breathing during respiratory distress.

Albumin Treatment

Albumin treatment is also often allotted to SCD patients experiencing TRALI [9,14,18]. This is particularly true when patients experience hypotension [18]. The presence of hypotension often results in a lack of response to intravenous fluid therapy, often provided as a supportive treatment protocol for TRALI [9]. In these cases, patients will often receive 5% albumin rather than saline to replace fluid loss [18].

Erythropoietin and Iron Use

When ongoing blood transfusion reactions are occurring, as seen with TRALI, erythropoietin and intravenous iron are often provided to patients. The goal of this type of treatment is to increase the red blood cell count and alleviate the onset of severe anemia [5]. This treatment is often provided with other supportive care modalities, including those listed in previous segments.

TRALI preventative options

Due to the lack of effective treatment options, attention has been placed on preventative measures aimed at preventing or mitigating the onset of TRALI. These include conducting blood antibody testing of donors, creating enhanced and standardized blood and plasma protocols, engaging in rapid reporting responses to blood banks, and the provision of rituximab as prophylaxis when appropriate [5,8-10]. Each of these modalities is briefly discussed below.

Blood Antibody Testing of Donors

One preventative measure that has been suggested includes an increased emphasis on the testing of donor blood and plasma [8,10]. This includes testing the donor blood for anti-leukocyte antibodies, which account for approximately 80% of TRALI cases [4]. Moreover, testing for anti-human leukocyte antigen (HLA) and anti-human neutrophil antigen (HNA) antibodies is also necessary due to their involvement in the development of TRALI [8]. In some cases, healthcare workers have argued that multiparous donations without leucocyte alloantibodies testing should not be used as well [9]. Though testing does occur at many facilities, it does not always include the testing of these features.

Enhanced and Standardized Blood and Plasma Selection Protocols

In addition to increasing testing in transfusion facilities, there has also been a push to enhance and standardize protocols for the selection of blood and plasma across the nation. Examples have been provided by both international protocols and facility protocols that are in place around the country. The United Kingdom utilizes male donors only due to the heightened increase in HLA/HNA antibodies. Women who have been previously pregnant are automatically disqualified from donation [10]. Some facilities within the United States have also excluded the use of fresh frozen plasma from female donors due to the heightened risk of TRALI development [16]. Regardless of these protocols, it is important to be consistent at a national level to ensure that standardized practices can be obtained.

Rapid Reporting to Blood Banks

Another standard that requires enhancement is the rapid reporting efforts to blood banks when donations cause adverse events such as TRALI. Once the blood bank receives the report they should test all donor samples for the presence of anti-HLA and anti-HNA antibodies [8]. This may provide the opportunity to dispose of the donor samples and inform other recipients to assist in ceasing its use in other patients [8]. Enhanced reporting protocols may be key to the future prevention of SCD-related TRALI.

Rituximab Prophylaxis

One final prevention and mitigation measure includes the use of rituximab as a preventive option. The rationale of this prophylaxis is intended for patients with a history of severe delayed hemolytic transfusion reactions. In addition to this preventative treatment, blood that is “least incompatible” should be sourced to continue the required blood transfusions for SCD patients [5].

Potential future treatments

Researchers and hematologists are constantly seeking improved treatment options to provide SCD patients with minimal adverse effects and enhance the treatment options of TRALI. Currently, the research and clinical testing process include the use of anti-CD40L monoclonal antibodies and immunotherapy [4,11,12]. Clinical trials for anti-CD40L are currently underway using rats. The studies and trials have produced positive results, and the use of this antibody has demonstrated success in preventing the onset of pulmonary edema in the TRALI mouse study [12]. Alternatively, research has indicated that the immune system plays a vital role in the onset of TRALI, making immunotherapy a focus of research [11]. One therapeutic approach currently being studied includes IL-10 therapy [4]. The goal of this therapy is to increase the immune-regulatory cytokine that is hindered during the transfusion process [11]. These emerging treatment modalities are demonstrating promising results for countering TRALI more effectively than existing modalities.

Limitations

This review includes studies from the past six years and reports prior to 2015 were not included to focus on the novel therapies of this complication. In addition, review articles and animal studies were included and study designs such as observational and other experimental studies were not included merely due to the limited reports available with no definite conclusion. Preclinical studies are conducted globally in this domain and more studies are yet to be reported.

## Conclusions

The onset of TRALI can have devastating impacts on patients receiving blood transfusions. The presence of SCD increases the risk of developing TRALI due to the dependency on transfusions that often accompany the hereditary disease. Despite studying SCD for over a century, few treatment and management options exist that effectively address the onset of TRALI. The provision of supportive care modalities, while helpful, falls short of the desire of hematologists and SCD patients alike. It is critical that new treatment options continue to be explored to identify better methods of prevention and treatment protocols related to TRALI. Moreover, to enhance prevention and mitigation strategies, blood and plasma testing and reporting protocols must be increased and standardized nationally. Prevention of the onset of TRALI may be the most effective treatment option for SCD patients who are dependent on blood transfusion for survival.
